The article "Extract of Spatholobus suberctus Dunn ameliorates ischemia-induced injury by targeting miR-494" was retracted in 2019. Reasons: concerns about the data; concerns about the images.

# Extract of *Spatholobus suberctus* Dunn ameliorates ischemia-induced injury by targeting miR-494

**DOI:** 10.1371/journal.pone.0184348

**Published:** 2017-09-07

**Authors:** Shiqing Song, Faliang Lin, Pengyan Zhu, Changyan Wu, Shuling Zhao, Qiao Han, Xiaomei Li

**Affiliations:** 1 Yantai Yuhuangding Hospital of Qingdao University Medical College, Yantai, Shandong, China; 2 Yantai Hospital of Traditional Chinese Medicine, Yantai, Shandong, China; 3 Yantai Blood Center, Yantai, Shandong, China; 4 Affiliated Hospital of Zunyi Medical College, Zunyi, Guizhou, China; Massachusetts General Hospital/Harvard Medical School, UNITED STATES

## Abstract

Cerebral stroke is a leading cause of death and permanent disability. The current therapeutic outcome of ischemic stroke (>85% of all strokes) is very poor, thus novel therapeutic drug is urgently needed. *In vitro* cell model of ischemia was established by oxygen-glucose deprivation (OGD) and in *vivo* animal model of ischemia was established by middle cerebral artery occlusion (MCAO). The effects of *Spatholobus suberctus* Dunn extract (SSCE) on OGD-induced cell injury, MCAO-induced neural injury and miR-494 level were all evaluated. The possible target genes were virtually screened utilizing bioinformatics and verified by luciferase assay. Subsequently, the effects of abnormally expressed miR-494 on OGD-induced cell injury and target gene expression were determined. Additionally, whether SSCE affected target gene expression through modulation of miR-494 was studied. Finally, the effects of aberrantly expressed Sox8 on OGD-induced injury and signaling pathways were estimated. SSCE reduced OGD-induced cell injury and ameliorated MCAO-induced neuronal injury, along with down-regulation of miR-494. Then, OGD-induced cell injury was increased by miR-494 overexpression but decreased by miR-494 silence. Sox8 was a target gene of miR-494, and SSCE could up-regulate Sox8 expression via down-regulating miR-494. Afterwards, OGD-induced cell injury was proved to be increased by Sox8 inhibition but reduced by Sox8 overexpression. Finally, OGD-induced inhibition of PI3K/AKT/mTOR and MAPK pathways was further inhibited by Sox8 silence but activated by Sox8 overexpression. SSCE ameliorates ischemia-induced injury both *in vitro* and *in vivo* by miR-494-mediated modulation of Sox8, involving activations of PI3K/AKT/mTOR and MAPK pathways.

## Introduction

Cerebral stroke, also termed stroke or cerebral vascular accident, is an acute cerebral vascular disease which includes multiple forms, such as ischemic stroke, subarachnoid hemorrhage and intracerebral hemorrhage [1]. It has been estimated to be the second most common cause of death by the Global Burden of Diseases, Risk Factors Study and Injuries in 2010, as well as the leading cause of adult long-term disability [2]. Ischemic stroke, accounting for more than 85% of all strokes, is caused by the occlusion of a major cerebral artery with a thrombus or an embolism, resulting in deprivation of glucose and oxygen as well as subsequent tissue death [3]. Approved by FDA, tissue plasminogen activator is the only effective drug for ischemic stroke [4]. Nevertheless, less than 7% of patients with acute stroke receive thrombolytic treatment due to the short therapeutic window and numerous exclusions [5]. Therefore, it appears to be urgent to explore alternative potential approaches for the improvement of stroke outcome.

Recently, Chinese herbal medicine has been reported to possess potential benefits for treatment of stroke [6]. *Spatholobus suberctus* Dunn is a common herbal medicine which has been widely used for treatment of blood deficiency, irregular menstruation and rheumatalgia in traditional Chinese and folk medicine [7]. In recent years, *Spatholobus suberctus Dunn* extract (SSCE) has been identified to possess reactive oxygen species scavenging capacity [8] and antineoplastic activity [9]. In addition, SSCE is also reported to inhibit osteoclast differentiation and bone loss induced by *Porphyromonas gingivalis* [10]. Even though the role of SSCE in the dissolution of stasis has been widely applied, the precise role of SSCE in stroke as well as the underlying molecular mechanism remains controversial.

MicroRNAs (miRs) are a class of small non-coding RNAs that could participate in modulation of target genes through pairing with 3’UTR in the mRNA of target gene [11]. Various miRs are proved to contribute to the cell death of acute ischemic stroke, such as miR-29b and miR-124 [12–14]. Ectopic expression of miR-494, which is located on chromosome 14q32.31, has been identified in diverse cancers, for example, lung cancer, brain cancer, liver cancer, *etc*. [15]. A recent literature by Welten *et al*. reported that repression of miR-494 could improve blood flow recovery after ischemia [16]. Thus, we hypothesized that miR-494 might be involved in the outcome of ischemia. PC12 cells, which are derived from the rat pheochromocytoma of medulla, have been widely used for establishing cell model of ischemic stroke in combination with oxygen-glucose deprivation (OGD) [17]. PC12 cells with OGD can simulate ischemic stroke and provide an adequate model for exploration of potential neuroprotective drugs [18]. Herein, we constructed ischemic stroke model in PC12 cells with OGD and explored the potential role of SSCE in the stroke. Moreover, the possible molecular mechanism involving in miR-494 and signaling pathways were also studied. Besides, the effects of SSCE on stroke were verified *in vivo*.

## Materials and methods

### Cell culture and OGD treatment

The PC12 cells (Kunming Institute of Zoology, Kunming, China) were maintained in Dulbecco’s Modified Eagles Medium (DMEM) containing 10% (v/v) fetal bovine serum, 100 U/mL penicillin and 100 μg/mL streptomycin (all from Gibco, Grand Island, NY, USA). Under normal conditions, cells were cultured in a humidified incubator at 37°C with 5% CO_2_. Under a condition of OGD, the culture medium was replaced by a glucose-free DMEM with or without SSCE, and cells were subjected into an anaerobic chamber which was equilibrated with a gas mixture of 5% CO_2_ and 95% N_2_ (v/v) for various time intervals.

### Extraction of *Spatholobus suberctus* Dunn

The dried *Spatholobus suberctus Dunn* herbs (2500 g) were cut into small pieces, soaked in Mili-Q (Millipore, Billerica, MA, USA) water for 1 h, and extracted under reflux for 2 h which was repeated twice. The solution was sieved on a 120 mesh-filter cloth and stored at 4°C overnight. Then, the supernatant was centrifuged, evaporated, and dried in a vacuum oven (0.01 Pa) at 60°C for 6 h. Dissolved in Mili-Q water, the crude extract was subjected to polyamide column chromatography, and eluted with 0%, 30% and 95% ethanol in turns. Fractions eluted with 30% ethanol were collected, evaporated and dried in a vacuum oven to obtain 13.89 g SSCE. Subsequently, SSCE was dissolved in dimethyl sulfoxide (DMSO) and the concentration was 1 g/mL. For the following experiments, SSCE was diluted with culture media to a final concentration of 5 μg/mL.

### Cell Counting Kit-8 (CCK-8) assay

Cell viability was measured by using a CCK-8 (Dojindo, Gaithersburg, MD, USA) in accordance with the supplier’s instructions. Briefly, cells were seeded into 96-well plates with a density of 5 × 10^3^ cells/well and cultured. After treatments, 10 μL of CCK-8 solution was added to each well and the mixture was incubated at 37°C for 1 h under normal condition. The absorbance at 450 nm was determined using a microplate reader (Bio-Rad, Hercules, CA, USA).

### Apoptosis assay

Cell apoptosis was estimated by Flow cytometry analysis following the protocol of Annexin V-FITC/propidium iodide (PI) apoptosis detection kit (Beijing Biosea Biotechnology, Beijing, China). Briefly, 1 × 10^5^ cells were seeded in each well of 6-well plates and cultured. After treatments, cells were collected, washed with cold phosphate-buffered saline (PBS) and resuspended in binding buffer. The cells were then stained with 10 μL Annexin V-FITC and 5 μL PI in the dark, followed by measurements with a flow cytometer (Beckman Coulter, Miami, FL, USA).

### miR transfection

miR-494 mimic, miR-494 inhibitor and their controls (mimic control and inhibitor control) were synthesized by GenePharma Co. (Shanghai, China). These miRs were transfected into PC12 cells using Lipofectamine 3000 reagent (Invitrogen, Carlsbad, CA, USA) following the manufacturer’s instructions.

### Transfection and generation of stably transfected cell lines

The full-length rat Sox8 sequences were sub-cloned into pEX-2 plasmid (GenePharma) to generate pEX-Sox8. Short-hairpin RNA directed against rat Sox8 were constructed into U6/GFP/Neo plasmid (GenePharma) to generate sh-Sox8. The empty pEX-2 plasmid and U6/GFP/Neo plasmid carrying a non-targeting sequence (sh-NC) were used as negative controls of pEX-Sox8 and sh-Sox8, respectively. These recombined plasmids were respectively transfected into PC12 cells by using Lipofectamine 3000 reagent (Invitrogen) following the manufacturer’s instructions. Culture medium supplemented with 0.5 mg/mL G418 (Sigma-Aldrich, St Louis, MO, USA) was used for selection of stably transfected cells. Approximately 4 weeks later, the PC12 cell lines with stable transfection (G418-resistant cells) were established.

### Quantitative reverse transcription PCR (qRT-PCR)

Trizol reagent and Ambion^®^ DNase I (both from Invitrogen) were used for extraction of total RNA according to the manufacturer’s protocol. On the basis of protocols of suppliers, Taqman MicroRNA Reverse Transcription Kit (for quantification of miR-494) and Multiscribe RT kit (for quantification of Sox8) (both from Applied Biosystems, Foster City, CA, USA) were used for reverse transcription. Then, quantitation of miR-494 and Sox8 was performed using Taqman Universal Master Mix II (Applied Biosystems) following the protocols of suppliers. Relative expression was calculated according to the 2^-ΔΔCt^ method [19], by normalizing to U6 (miR-494) and GAPDH (Sox8) expression levels, respectively. The Primers were shown in S1 Table.

### Dual luciferase activity assay

Fragments of wild-type rat Sox8 3’UTR containing the putative miR-494-binding sites were sub-cloned into the pmirGLO vector (Promega, Madison, WI, USA), and the resultant plasmid was referred to as Sox8-WT. The recombined Sox8-WT was served as a template for site-mutation using Directed Mutagenesis System (Invitrogen) to generate Sox8-Mut. Then, cells were co-transfected with Sox8-WT (Sox8-Mut) and miR-494 mimic (mimic control) using Lipofectamine 3000 reagent (Invitrogen), followed by estimation of luciferase activity using the dual-luciferase assay system (Promega) in accordance with the manufacturer’s information.

### Western blot analysis

The protein of cells was extracted using RIPA lysis buffer (Beyotime Biotechnology, Shanghai, China) supplemented with phosphatase inhibitor cocktail (Sigma-Aldrich) and protease inhibitor cocktail (Roche, Indianapolis, IN, USA). After quantification with the BCA™ Protein Assay Kit (Pierce, Appleton, WI, USA), equivalent proteins were separated by 10% sodium dodecyl sulfate-polyacrylamide gel electrophoresis (SDS-PAGE). Then, proteins in the gels were transferred to polyvinylidene difluoride (PVDF) membranes (Millipore), and the membranes were blocked by 5% skim milk. After washing, membranes were incubated at 4°C overnight with primary antibodies against B cell lymphoma-2 (Bcl-2, ab196495), Bcl-2-associated X protein (Bax, ab182733), pro caspase-3 (ab90437), cleaved caspase-3 (ab49822), phosphatidylinositol-3-kinase (PI3K, ab191606), phosphorylated PI3K (p-PI3K, ab182651), GAPDH (ab181603) (all from Abcam, Cambridge, UK), pro caspase-9 (9508), cleaved caspase-9 (9507), AKT (9272), phosphorylated AKT (p-AKT, 9271), mechanistic target of rapamycin (mTOR, 2972), phosphorylated mTOR (p-mTOR, 2971), mitogen-activated protein kinase (MAPK, 9212), phosphorylated MAPK (p-MAPK, 9211) (all from Cell Signaling Technology, Beverly, MA, USA) or Sox8 (sc-374445, Santa Cruz, Santa Cruz, CA, USA). After washing again, the membranes were incubated with secondary antibodies marked by horseradish peroxidase for 1 h at room temperature. The PVDF membranes were washed and reacted with an enhanced chemiluminescence (ECL) system (Amersham Biosciences, Piscataway, New Jersey, USA). The signals were captured and detected using Image Lab™ software (Bio-Rad), and the intensity of bands was analyzed using Image J software (version 1.46; National Institutes of Health, Bethesda, MD, USA).

### Surgical procedure and grouping of rats

Middle cerebral artery occlusion (MCAO) was carried out for construction of stroke model in rats as described previously [20]. In brief, after anesthetization, the right common (CCA), right external (ECA) and right internal (ICA) carotid arteries were exposed and a nylon suture was inserted into CCA and advanced up to the origin of the MCA. Ischemic occlusion was confirmed by a laser Doppler flowmeter (Perimed, Jarfalla, Sweden), showing a reduction of >70% of baseline. After 1 h of occlusion, reperfusion was done via withdrawal of the nylon suture. The procedure was approved by the Ethics Committee of the Yantai Yuhuangding Hospital of Qingdao University Medical College. A total of 50 male adult Sprague-Dawley rats weighing 250-300g (Shanghai Science Academy animal center, Shanghai, China) were randomly assigned into five groups (n = 10 for each group), including Sham, MCAO, MCAO+SSCE (L), MCAO+SSCE (M) and MCAO+SSCE (H) groups. Rats in sham group were received an identical procedure without occlusion. Rats in MCAO+SSCE groups were received MCAO surgery along with SSCE (once a day by gavage) at doses of 20 mg/kg (L), 40 mg/kg (M) and 80 mg/kg (H).

### Modified neurological severity scores (mNSSs)

Neurological deficits were assessed using mNSSs at 2, 5, 8, 11, or 14 days post-MCAO as described previously [21]. In brief, a blinded assessor scored the neurological deficits of rats on the basis of an 18-point scale. The score of 0 was referred to as normal and the score of 18 was referred to as maximal deficit.

### Rota-rod test

Motor coordination and learning ability was evaluated by rota-rod test as described previously [21]. A day before surgery, rats received a training on a rota-rod apparatus (diameter 6.0 cm, Ugo Basile, Milano, Italy) with a constant speed at 3 rpm until they could remain on the rotating spindle for 180 s. The measurements with a spindle speeds of 5 rpm and 15 rpm were performed at 2, 5, 8, 11, and 14 days post-MCAO, and the residence times on the spindle were recorded. Rats were rested for 1 h between two trials.

### Infarct volume assessment

After 14 days of maintaining, rats were sacrificed and the whole brains were separated and cut into 2-mm slices coronally. Subsequently, the brain slices were incubated in 2% 2, 3, 5-triphenyltetrazolium chloride (TTC; Sigma-Aldrich) at 37°C for 30 min in the dark, and then fixed with 4% paraformaldehyde. The infarct volume was analyzed by Image J software and was calculated by multiplying infarct areas by thickness. Besides, the infarct areas were normalized through multiplying measured areas by ipsilateral to contralateral hemisphere area ratios.

### Statistical analysis

All experiments were repeated three times. The results of multiple experiments were presented as the mean ± standard error of the mean (SEM). Statistical analysis was performed using Graphpad Prism 5 software (GraphPad, San Diego, CA, USA). The *P*-values were calculated using the one-way analysis of variance (ANOVA) with post hoc Bonferroni’s correction. A *P*-value of <0.05 was considered to indicate a statistically significant result.

## Results

### OGD induced cell injury in PC12 cells

Cell viability and apoptosis were assessed at 0, 2, 4, 6 and 8 h post-OGD. When the OGD lasted for 4 h or longer, cell viability was markedly decreased compared with non-treated cells (*P* < 0.05, *P* < 0.01 or *P* < 0.001, **Fig 1A**). Conversely, percentages of apoptotic cells were significantly elevated by 2 h, 4 h (both *P* < 0.05), 6 h and 8 h (both *P* < 0.001) of OGD treatments (**Fig 1B and S1 Fig**). Meantime, the pro-apoptotic Bax, active caspase-3 and active caspase-9 were all up-regulated gradually as the increasing of OGD duration, whereas anti-apoptotic Bcl-2 showed the opposite trend (**Fig 1C and 1D**). Results illustrated that OGD could induce cell injury in PC12 cells, and the duration of OGD was 6 h for the subsequent experiments.

**Fig 1:** Oxygen and glucose deprivation (OGD) reduces cell viability but promotes cell apoptosis in PC12 cells. **A.** Cell viability by Cell Counting Kit-8 assay. **B.** Cell apoptosis by flow cytometry. **C-D.** Protein expression of apoptosis-associated proteins by Western blot analysis. Data are presented as the mean ± standard error of the mean (SEM). *, *P* < 0.05; **, *P* < 0.01; ***, *P* < 0.001. Bcl-2, B cell lymphoma-2; Bax, Bcl-2-associated X protein; P-, pro; C-, cleaved; C/P-, cleaved/pro.

### Preconditioning with SSCE protected PC12 cells against OGD-induced injury

Cell viability was markedly reduced with the presence of 10–20 μg/μl SSCE (*P* < 0.05 or *P* < 0.001) whereas the reduction under 5 μg/μl SSCE was non-significant, indicating the maximal dose of SSCE was 5 μg/μl (**Fig 2A**). Results in **Fig 2B** showed the decreased cell viability induced by OGD was remarkably increased by 2–5 μg/μl SSCE preconditioning compared with OGD group (*P* < 0.05). Oppositely, the increased cell apoptosis induced by OGD was significantly reduced by 2–5 μg/μl SSCE preconditioning compared with OGD group (*P* < 0.05 or *P* < 0.01, **Fig 2C and S2 Fig**). Meantime, the OGD-induced alterations of apoptosis-associated proteins at protein level were all significantly decreased by 2–5 μg/μl SSCE preconditioning (**Fig 2D and 2E**). The effects of 1 μg/μl SSCE on OGD-induced injury were non-significant. The results indicated that preconditioning with SSCE protected PC12 cells against OGD-induced injury in a dose-dependent manner.

**Fig 2:** Oxygen and glucose deprivation (OGD)-induced cell injury is attenuated by *Spatholobus suberctus* Dunn extract (SSCE). **A-B.** Cell viability by Cell Counting Kit-8 assay. **C.** Cell apoptosis by flow cytometry. **D-E.** Protein expression of apoptosis-associated proteins by Western blot analysis. Data are presented as the mean ± SEM. *, *P* < 0.05; **, *P* < 0.01; ***, *P* < 0.001. Bcl-2, B cell lymphoma-2; Bax, Bcl-2-associated X protein; P-, pro; C-, cleaved; C/P-, cleaved/pro.

### SSCE reduced infarct volume and improved neurological deficits and motor impairments

Next, the *in vivo* effects of SSCE on rats with MCAO were further evaluated. After 14 days of maintaining, there was nearly no infarct volume in the brain slices of sham group whereas that of the MCAO group was approximately 140 mm^3^ (**Fig 3A**). Compared with the MCAO group, infarct volume was significantly reduced by 20 mg/kg SSCE (*P* < 0.05), 40 mg/kg SSCE (*P* < 0.01) and 80 mg/kg SSCE (*P* < 0.01). Likewise, the mNSSs of rats in the Sham group were nearly zero whereas that in the MCAO group was about 7–10 at 2–14 days post-MCAO (**Fig 3B**). The mNSSs was markedly reduced by the treatments of SSCE at 2–14 days post-MCAO (*P* < 0.05 or *P* < 0.01). In addition, the residence times on the spindle at both 5 and 15 rpm were significantly reduced by MCAO compared with the Sham group (*P* < 0.001, **Fig 3C and 3D**). Administration of SSCE markedly prolonged the residence times at 2–14 days post-MCAO compared with the MCAO group (*P* < 0.05, *P* < 0.01 or *P* < 0.001). Results indicated that SSCE reduced infarct volume and improved neurological deficits and motor impairments.

**Fig 3:** *Spatholobus suberctus* Dunn extract (SSCE) reduces infarct volume and improves neurological deficits and motor impairments. Rats were randomly assigned into five groups. Doses of SSCE were 20 mg/kg (L), 40 mg/kg (M) and 80 mg/kg (H). **A.** Infarct volume by 1% 2,3,5-triphenyl tetrazolium chloride (TTC) staining. **B.** Modified neurological severity scores (mNSSs). Rota-rod test at spindle speeds of 5 rpm **(C)** and 15 rpm **(D).** Data are presented as the mean ± SEM (A-B) or mean + SEM. * indicates significant differences compared with the MCAO group. *, *P* < 0.05; **, *P* < 0.01; ***, *P* < 0.001. # indicates significant differences compared with the Sham group. ###, *P* < 0.001. MCAO, middle cerebral artery occlusion.

### SSCE down-regulated miR-494 in PC12 cells

Subsequently, we explored the change of miR-494 in PC12 cells during OGD. Expression of miR-494 was significantly up-regulated at 4 h (*P* < 0.05), 6 h and 8 h (both *P* < 0.01) post-OGD (**Fig 4A**). Data in **Fig 4B** showed the OGD induced up-regulation of miR-494 was reversed by SSCE preconditioning compared with the OGD group (*P* < 0.01), indicating SSCE could down-regulate miR-494 in PC12 cells during OGD.

**Fig 4:** MicroRNA (miR)-494 is up-regulated by oxygen and glucose deprivation (OGD) but the up-regulation is reversed by *Spatholobus suberctus* Dunn extract (SSCE). mRNA expression of miR-494 was determined by quantitative reverse transcription PCR (qRT-PCR). **A.** miR-494 level at 0, 2, 4, 6, 8 h post-OGD. **B.** miR-494 level after treatments of OGD and SSCE. Data are presented as the mean ± SEM. *, *P* < 0.05; **, *P* < 0.01.

### OGD-induced injury was increased by miR-494 overexpression but was reversed by miR-494 inhibition

To explore the influence of miR-494, miR-494 was aberrantly expressed in PC12 cells via cell transfection. In **Fig 5A**, miR-494 was significantly up-regulated in cells transfected with miR-494 mimic compared with the mimic control group while was dramatically down-regulated in cells transfected with miR-494 inhibitor compared with the inhibitor control group (both *P* < 0.01), suggesting miR-494 was abnormally expressed after transfection. CCK-8 assay showed OGD-induced decreases of cell viability were further decreased by miR-494 overexpression but were elevated by miR-494 inhibition when compared to respective controls (both *P* < 0.05, **Fig 5B**). Conversely, OGD-induced elevation of cell apoptosis was further increased by miR-494 overexpression while was decreased by miR-494 silence when compared to respective controls (both *P* < 0.05, **Fig 5C and S3 Fig**). Moreover, the alterations of apoptosis-associated proteins induced by OGD were significantly increased by miR-494 overexpression (*P* < 0.05 or *P* < 0.01) but were reduced by miR-494 inhibition (*P* < 0.01 or *P* < 0.001, **Fig 5D and 5E**). Taken together, we concluded that abnormal expression of miR-494 affected OGD-induced cell injury in PC12 cells.

**Fig 5:** Oxygen and glucose deprivation (OGD)-induced cell injury is attenuated by microRNA (miR)-494 silence but aggravated by miR-494 overexpression. **A.** miR-494 level by quantitative reverse transcription PCR (qRT-PCR). **B.** Cell viability by Cell Counting Kit-8 assay. **C.** Cell apoptosis by flow cytometry. **D-E.** Protein expression of apoptosis-associated proteins by Western blot analysis. Data are presented as the mean ± SEM. *, *P* < 0.05; **, *P* < 0.01. Bcl-2, B cell lymphoma-2; Bax, Bcl-2-associated X protein; P- pro; C-, cleaved.

### miR-494 negatively correlated with Sox8 expression

Predicted by bioinformatics, Sox8 was supposed to be a target of miR-494. First of all, the expression of Sox8 in OGD-treated PC12 cells was estimated. Results in **Fig 6A** showed Sox8 mRNA expression was significantly down-regulated at 4 h (*P* < 0.05), 6 h (*P* < 0.01) and 8 h (*P* < 0.001) post-OGD, which was opposite to the alteration of miR-494. In **Fig 6B–6D**, mRNA and protein levels of Sox8 were observably reduced by miR-494 overexpression but were significantly increased by miR-494 inhibition when compared with respective controls (*P* < 0.05 or *P* < 0.01), suggesting that miR-494 could negatively regulate Sox8 expression. The following luciferase assay verified the direct interaction between miR-494 and Sox8 3’UTR, presenting that luciferase activity was markedly reduced by co-transfection with Sox8-WT and miR-494 mimic compared with co-transfection with Sox8-WT and mimic control (*P* < 0.05) whereas the difference between co-transfections with Sox8-Mut was non-significant (**Fig 6E**). Therefore, we were suggestive of negative regulations between miR-494 and Sox8.

**Fig 6:** Sox8 is a target gene of microRNA (miR)-494. **A-B.** mRNA level of Sox8 by quantitative reverse transcription PCR (qRT-PCR). **C-D.** Protein level of Sox8 by Western blot analysis. **E.** Relative luciferase activity by luciferase assay. Data are presented as the mean ± SEM. *, *P* < 0.05; **, *P* < 0.01; ***, *P* < 0.001. Sox8-WT, pmirGLO vector containing fragments of wild-type rat Sox8 3’UTR; Sox8-Mut, mutant Sox8-WT.

### SSCE up-regulated Sox8 through down-regulating miR-494

To identify whether SSCE affected expression of Sox8 through modulating miR-494, cells transfected with mimic control or miR-494 were treated with OGD and SSCE. In **Fig 7A–7C**, OGD obviously decreased expression of Sox8 compared with the control group (*P* < 0.01), whereas the down-regulation of Sox8 was remarkably increased by SSCE preconditioning compared with the OGD group (*P* < 0.01 or *P* < 0.001). Moreover, the SSCE induced up-regulation of Sox8 was dramatically decreased by miR-494 overexpression compared with the mimic control+OGD+SSCE group (*P* < 0.01 or *P* < 0.001). All the results implied SSCE up-regulated Sox8 through down-regulating miR-494.

**Fig 7:** *Spatholobus suberctus* Dunn extract (SSCE) up-regulates Sox8 by down-regulating microRNA (miR)-494. **A.** Sox8 mRNA level by quantitative reverse transcription PCR (qRT-PCR). **B-C.** Sox8 protein level by Western blot analysis. Data are presented as the mean ± SEM. **, *P* < 0.01; ***, *P* < 0.001. OGD, oxygen and glucose deprivation.

### OGD-induced injury was reduced by Sox8 overexpression but was increased by Sox8 silence

To figure out the influence of Sox8 on PC12 cells with OGD, stably transfected cell lines were constructed. As evidence from **Fig 8A–8C**, both mRNA and protein expression of Sox8 were obviously elevated in pEX-Sox8 transfected cells (*P* < 0.01 or *P* < 0.001) but were significantly reduced in sh-Sox8 transfected cells compared with respective controls (*P* < 0.01). When compared to pEX-2 group, OGD-induced decrease of cell viability as well as OGD-induced increase of cell apoptosis were both attenuated markedly (*P* < 0.05 or *P* < 0.01) by Sox8 overexpression, whereas the effects of Sox8 inhibition on cell viability and apoptosis were just the opposite (**Fig 8D and 8E and S4 Fig**). Additionally, the changes of apoptosis-associated proteins induced by OGD were further increased by Sox8 inhibition while were reversed by Sox8 overexpression (**Fig 8F and 8G**). As a consequence, we concluded that OGD-induced injury could be decreased by Sox8 overexpression but was increased by Sox8 silence.

**Fig 8:** Oxygen and glucose deprivation (OGD)-induced cell injury is attenuated by Sox8 overexpression but aggravated by Sox8 silence. **A.** Sox8 mRNA level by quantitative reverse transcription PCR (qRT-PCR). **B-C.** Sox8 protein level by Western blot analysis. **D.** Cell viability by Cell Counting Kit-8 assay. **E.** Cell apoptosis by flow cytometry. **F-G.** Protein expression of apoptosis-associated proteins by Western blot analysis. Data are presented as the mean ± SEM. *, *P* < 0.05; **, *P* < 0.01; ***, *P* < 0.001. Bcl-2, B cell lymphoma-2; Bax, Bcl-2-associated X protein; P-, pro; C-, cleaved; pEX-Sox8, pEX-2 plasmid carrying full-length rat Sox8 sequences; sh-Sox8, U6/GFP/Neo plasmid carrying short-hairpin RNA directed against rat Sox8; sh-NC, U6/GFP/Neo plasmid carrying a non-targeting sequence.

### Sox8 overexpression decreased OGD-induced injury by activation of PI3K/AKT/mTOR and MAPK pathways

To reveal the underlying mechanisms of Sox8-associated regulations, the phosphorylation of key kinases involved in PI3K/AKT/mTOR and MAPK pathways was evaluated. Western blotting results showed phosphorylation levels of PI3K, AKT, mTOR and MAPK were all significantly reduced by OGD treatment (*P* < 0.01, **Fig 9A–9D**). Meanwhile, the OGD-induced reduction of these phosphorylated kinases was reversed by Sox8 overexpression (*P* < 0.001) but was further reduced by Sox8 inhibition (*P* < 0.01), indicating that abnormal expression of Sox8 affected OGD-induced injury by modulation of PI3K/AKT/mTOR and MAPK pathways.

**Fig 9:** Oxygen and glucose deprivation (OGD) induced inhibition of PI3K/AKT/mTOR and MAPK pathways are further inhibited by Sox8 silence but are reversed by Sox8 overexpression. Phosphorylation levels of key kinases involved in PI3K/AKT/mTOR **(A-B)** and MAPK **(C-D)** pathways were determined by Western blot analysis. Data are presented as the mean ± SEM. **, *P* < 0.01; ***, *P* < 0.001. pEX-Sox8, pEX-2 plasmid carrying full-length rat Sox8 sequences; sh-Sox8, U6/GFP/Neo plasmid carrying short-hairpin RNA directed against rat Sox8; sh-NC, U6/GFP/Neo plasmid carrying a non-targeting sequence; PI3K, phosphatidylinositol-3-kinase; mTOR, mechanistic target of rapamycin; MAPK, mitogen-activated protein kinase; p-, phosphorylated.

## Discussion

Stroke is not only a major cause of mortality but also a leading reason of permanent disability worldwide [22]. The outcome of ischemic stroke, majority of all strokes, remains very poor although mounting studies have identified various neuroprotective agents. Thus, more studies should be focused on the exploration of effective therapeutic drugs for ischemic stroke. In our study, we established cell model and animal model of ischemic stroke and interestingly identified SSCE could decrease OGD-induced cell injury, reduced infarct volume and improved neurological deficits and motor impairments. Then, miR-494 was found to be up-regulated after OGD treatment but down-regulated by SSCE preconditioning. Following experiments proved that abnormally expressed miR-494 affected OGD-induced cell injury by targeting Sox8 expression. Not surprisingly, the aberrantly expressed Sox8 was also proved to modulate OGD-induced cell injury. Moreover, PI3K/AKT/mTOR and MAPK pathways were involved in OGD treatment and the protective effect of Sox8 on OGD-induced cells.

The neuroprotective effects of SSCE on ischemic stroke were verified both *in vitro* and *in vivo*. Overwhelming evidence suggests cell death was observed and considered as the predominant phenomenon of ischemia-induced damage [23, 24]. In our study, OGD-induced decrease of cell viability and increase of cell apoptosis were all decreased by 2–5 μg/μl SSCE, suggesting the neuroprotective roles of SSCE *in vitro*. *In vivo* model of ischemic stroke was constructed through MCAO, by which the infarct volume was produced and the neurological deficits and motor impairments were observed. Administration of SSCE in rats effectively reduced infarct volume and improves neurological deficits and motor impairments, suggesting the neuroprotective roles of SSCE *in vivo*.

A literature demonstrated miR-494 suppression decrease carotid artery atherosclerotic lesion, suggesting a potential reduction of the ischemic stroke risk [25]. Results in our study stated miR-494 was up-regulated after OGD and the up-regulation could be reversed by SSCE treatment, indicating that miR-494 was associated with the protective effect of SSCE on OGD-induced injury. Subsequently, the specific effects of aberrantly expressed miR-494 on OGD-induced PC12 cells were verified. Results stated that OGD-induced reduction of cell viability was further decreased whereas OGD-induced enhancement of cell apoptosis was further increased by miR-494 overexpression. The inhibition on cell viability and the promotion on cell apoptosis of miR-494 in our study were consistent with previous studies [26, 27].

In common, miRs function through binding to 3’UTR of target genes, thus we screened the possible target genes of miR-494 by TargetScan virtually. Sex determining region Y-related high mobility group box (Sox) family proteins are involved in multiple pathological and physiological processes, including tumor progression [28, 29]. Sox8 has been reported as the target gene of miR-124 and suppresses cell proliferation in non-small lung cell carcinoma [30]. Another study also proved that Sox8 is a oncogenic gene in hepatocellular carcinoma [31]. Thus, we hypothesized Sox8 might affect cell proliferation and apoptosis of PC12 cells and thereby affect OGD-induced cell injury. As a consequence, we focused on the Sox8 among those screened target genes of miR-494. Results in our study illustrated that Sox8 was negatively regulated by miR-494, making us confirm Sox8 was a target gene of miR-494. The subsequent luciferase activity assay also consolidated the conclusion.

Afterwards, miR-494 was aberrantly expressed in PC12 cell, and the transfected cells were treated with OGD+SSCE in order to verify whether SSCE regulated Sox8 expression through regulating miR-494. Results in our study illustrated that SSCE could reverse OGD-induced down-regulation of Sox8, and the effect of SSCE could be abrogated be miR-494 overexpression, meaning that SSCE could regulate Sox8 expression through modulating miR-494. In addition, we performed additional experiments to fully verify the effect of abnormally expressed Sox8 on PC12 cell with OGD treatment. In detail, the decrease of cell viability induced by OGD was further reduced by Sox8 silence but reversed by Sox8 overexpression, and the increase of cell apoptosis induced by OGD was further enhanced by Sox8 silence but reversed by Sox8 overexpression. Therefore, Sox8 was identified to reduce OGD-induced cell injury by affecting cell viability and apoptosis, which was consistent with previous studies [30, 32].

Accumulating evidence has proved that PI3K/AKT/mTOR and MAPK signaling pathways are closely related to cell proliferation and apoptosis [33, 34]. PC12 cell apoptosis, induced by sodium nitroprusside or β-amyloid, has been reported to be repressed through PI3K/AKT/mTOR pathway [35, 36]. Likewise, cell apoptosis of PC12 cells could be suppressed by nobiletin [37] or gastrodin [38] through MAPK signaling pathway. Hence, to reveal underlying mechanism of SSCE modulation, the phosphorylation levels of key kinases involved in PI3K/AKT/mTOR and MAPK pathways were determined in PC12 cells with aberrantly expressed Sox8. Results in our study proposed that these two pathways were inhibited by OGD and further inhibited by Sox8 silence, while was activated by Sox8 overexpression. Therefore, activations of these two signaling pathways were involved in Sox8-mediated protection against OGD-induced injury in PC12 cells.

Collectively, SSCE was interestingly identified to improve ischemia-induced neuronal injury both *in vitro* and *in vivo*, and the protective effects were associated with miR-494. Further studies proved that the SSCE functioned through down-regulation of miR-494 by targeting Sox8, involving in activation of PI3K/AKT/mTOR and MAPK pathways. This study illustrated the potential role of SSCE in ischemic stroke and explained the underlying molecular mechanism, providing the theoretical basis for the traditional therapy with Chinese herbs.

## Supporting information

S1 Table Primers sequences. (DOCX)

S1 Fig Cell apoptosis after oxygen-glucose deprivation (OGD) for 0, 2, 4, 6, 8 h. (TIF)

S2 Fig Cell apoptosis after oxygen-glucose deprivation (OGD) along with Spatholobus suberctus Dunn extract (SSCE) treatments. (TIF)

S3 Fig Cell apoptosis after oxygen-glucose deprivation (OGD) and aberrant expression of miR-494. (TIF)

S4 Fig Cell apoptosis after oxygen-glucose deprivation (OGD) and aberrant expression of Sox8. (TIF)
